RETRACTED

# Spider Eye Development Editing and Silk Fiber Engineering Using CRISPR‐Cas

**DOI:** 10.1002/anie.202502068

**Published:** 2025-05-08

**Authors:** Edgardo Santiago‐Rivera, Thomas Scheibel

**Affiliations:** ^1^ Department of Biomaterials University of Bayreuth Prof.‐Rüdiger‐Borman Strasse 1 95448 Bayreuth Germany; ^2^ Bayreuth Zentrum für Kolloide und Grenzflächen Universität Bayreuth 95440 Bayreuth Germany; ^3^ Bayreuth Zentrum für Molekulare Biowissenshaften Universität Bayreuth 95440 Bayreuth Germany; ^4^ Bayreuther Materialzentrum Universität Bayreuth 95440 Bayreuth Germany; ^5^ Bayerisches Polymerinstitut University of Bayreuth 95440 Bayreuth Germany

**Keywords:** Eye‐loss, Fluorescent silk fibers, Genotype, Knock‐in, Knock‐out, Major ampullate silk

## Abstract

CRISPR‐Cas9 gene editing represents an effective and precise technology to induce mutations in the genome, and it has been applied to a wide range of organisms for diverse purposes. However, CRISPR‐based gene editing in spiders has not been reported to date. In this study, we demonstrate CRISPR‐mediated microinjection in parental spiders leading to both knock‐out (KO) and knock‐in (KI) mutations within the spider's offspring. The KO of the gene *sine oculis* causes total eye loss, confirming the role of the gene in the development of all spider eyes. The KI of a monomeric red fluorescent protein (mRFP‐KI) within a spider silk gene encoding one compound of the major ampullate silk of the spider *Parasteatoda tepidariorum* yields red fluorescent silk fibers. This finding demonstrates the feasibility of functionalizing silk proteins in spiders using CRISPR‐based gene editing without influencing silk assembly. Our study expands the application of CRISPR to spiders and provides insights in the fields of developmental genetics as well as material sciences.

## Graphical abstract

Spiders exhibit unique traits with significant implications for a diversity of fields, and gene editing provides new opportunities for advancing research in these areas. In this study, we developed a CRISPR‐Cas9 protocol for spiders, enabling gene knock‐outs/knock‐ins to study gene function and introduce new phenotypic traits.

## Introduction

During the last decade, the gene editing tool CRISPR‐Cas9 (clustered regularly interspaced short palindromic repeats and CRISPR‐associated protein 9) has revolutionized the field of biology.^[^ ^1^, ^2^ ^]^ The Cas9 protein contains two endonuclease domains capable of inducing a double‐stranded break (DSB) at a specific DNA target region. The protein binds to a single‐stranded RNA (ssRNA) known as the guide RNA (gRNA), whose sequence is designed to be complementary to the target region next to the protospacer adjacent motif (PAM), inducing the DSB.^[^ ^3^ ^]^ After the DSB, cells have two main alternative pathways to repair the DNA. The first and least precise is the nonhomologous end joining (NHEJ), which occurs when the two cleaved DNA strands are bound together, usually with mutations impairing the normal function of the protein. The second and more precise repair mechanism is termed homology‐directed repair (HDR), in which the homologous chromosome is used as a template to recover the cleaved area. The NHEJ is usually utilized to induce a gene knock‐out (KO) as it allows the introduction of errors that affect the gene of interest causing, for example, a premature stop codon or a miss‐sense in translation resulting in an unfinished or truncated protein with reduced or total loss of function, helping to characterize the role of a protein (Figure 1a). On the other hand, the HDR is used for knock‐in (KI) of a specific sequence by using the homologous chromosome or by the addition of a donor template. In the case of a donor template, the KI sequence is flanked by complementary sequences to the target region, misleading the repair mechanism into believing it is the homologue chromosome and driving the desired sequence to be copied from the donor into the intended genomic DNA sequence^[^ ^4^ ^]^ (Figure 1a). Because of its efficacy, CRISPR has been applied in a wide range of studies in developmental and evolutionary biology^[^ ^5^, ^6^, ^7^ ^]^ and for diverse applications such as in material sciences,^[^ ^8^, ^9^ ^]^ pest control,^[^ ^10^, ^11^ ^]^ and agriculture.^[^ ^12^, ^13^ ^]^ Considering the broad utilization in different scientific disciplines, it is, however, surprising that there is no report on spider‐related CRISPR applications.

RETRACTED

**Figure 1:** CRISPR‐Cas9 induced genetic modifications in spiders. a) The Cas9 protein binds to a designed guide RNA (gRNA) being complementary to the target region of the genome of the spider.^[^ ^1^, ^2^ ^]^ The resulting ribonucleoprotein (RNP) complex then binds to the complementary DNA strand in the genome, inducing a double‐strand break (DSB) near the protospacer‐adjacent motif (PAM) region.^[^ ^3^ ^]^ In principle, this cleavage can be repaired through either nonhomologous end‐joining (NHEJ) or homologous direct repair (HDR). b) Spiders were anesthetized with CO_2_ to prevent movement during injection. They were held by hand under the stereomicroscope while the loaded capillary needle was inserted into the lateral side of the opisthosoma to deliver the RNP solution, avoiding vital organs. Afterward, males were introduced for fertilization. Finally, the eggs were collected and reared. c) The gRNAs were either designed to knock‐out (KO) the eye development gene *sine oculis* (C1) or to target the spider silk gene *major ampullate spidroin 2* to induce a knock‐in (KI) of the gene encoding the monomeric red fluorescent protein (mRFP) (C2).

Remarkably, the evolutionary success of spiders hinges on the exceptional traits they possess, which not only offer valuable insights into a wide range of scientific questions but also underscore their significance as a research subject.^[^ ^14^, ^15^, ^16^ ^]^ Several factors contribute to the underrepresentation of spiders in research: first, they are a diverse group, and it is difficult to account for every single species^[^ ^17^ ^]^; second, because of their genome architecture, including genome duplication^[^ ^18^ ^]^; third, due to their cannibalistic nature, having to rear them individually, which, combined with other challenges, complicates their study.^[^ ^16^ ^]^ All these factors result in spiders being underrepresented in laboratory research compared to other arthropods such as mosquitoes^[^ ^11^ ^]^ and cockroaches.^[^ ^19^ ^]^

Nonetheless, recent advancements in developmental and genetic research in spiders have allowed the establishment of the cobweb spider *Parasteatoda tepidariorum* and the tiger bromeliad spider *Cupiennius salei* as research models in the study of spider biology under controlled laboratory conditions.^[^ ^16^, ^20^ ^]^ This body of research is important as spiders are among the most distant group to the subphylum of hexapoda within the arthropods,^[^ ^21^ ^]^ thus providing interesting evolutionary and developmental comparisons. For example, spiders have a remarkable unique ontogeny with different cell migration and other traits, including early cellularization and a short syncytial stage,^[^ ^16^, ^22^ ^]^ making them a remarkable model to study cell‐to‐cell communication and interaction during early ontogenesis. Therefore, we underline that the development of a gene editing tool within the order Araneae is important to elucidate the specific function of genes in relation to phenotypic traits during development, and more importantly, those that form in mid‐to‐late nymph stages that cannot be studied otherwise. Furthermore, Araneae are most famous for their silk, which is one hallmark fiber in the field of material sciences.^[^ ^23^, ^24^ ^]^ Successful spider silk engineering in vivo will, therefore, help to develop and employ new fiber functionalities for a broad range of applications. So far, genetic modifications in spiders have been only aimed at evolutionary and developmental research. These have been limited to RNA‐interference (RNAi) experiments, which are constrained by the spatiotemporal limitations of gene expression. Since the spider *P. tepidariorum* was recently established as a research archetype for studying spider biology,^[^ ^25^, ^26^, ^27^, ^28^ ^]^ it is a great model to develop CRISPR gene editing.

RETRACTED

## Results and Discussion

Wondering why CRISPR‐Cas9 gene editing has apparently so far not been used in spiders, we wanted to find out about the challenges behind this endeavor. After several failed setups, we investigated CRISPR‐Cas9 editing upon microinjecting the CRISPR solution into the hemolymph of adult female spiders of *P. tepidariorum* reaching their ovaries and mutating their offspring. The spiders were anesthetized with CO_2_ to prevent them from moving, while the procedure was carried out. The spiders were then held by hand under the stereomicroscope, while the loaded capillary needle was injected at the lateral side of the abdomen to deliver ∼2 µL of microinjection solution containing Cas9:gRNA (1 µg µL^−1^:800 ng∼1 µg µL^−1^) (Figure 1b). The microinjected solution tackled a spider's oocytes before it was mated with a male counterpart. This procedure allowed us to establish a protocol for implementing CRISPR‐based KO and KI gene editing in spiders. The prime target was the modification of spider silk (Figure 1c), namely the major ampullate silk gene *major ampullate spidroin‐2* (*masp2*). But due to the difficulties with establishing the CRISPR‐Cas9 technology in spiders, we first chose a simple‐to‐trace KO gene, namely *sine oculis* (*so*) also known as *Sox1* and *soA* (Figure 1c). The gene *so* regulates eye development in spiders but is not necessary for survival, and a KO of *so* should, therefore, lead to easy detectable phenotypes.

### CRISPR‐Induced Gene Knock‐Out (KO)

The gene *so* was previously identified through comparative evolutionary developmental studies in arachnids and is responsible for the development of all the eyes (Figure 2a).^[^ ^25^, ^26^, ^29^, ^30^ ^]^ Correspondingly, it was chosen for the CRISPR‐KO experiment because a mutation of this gene will cause a strong phenotype, helping to screen any mutation within the offspring.^[^ ^25^ ^]^ Offspring were analyzed using optical screening for the absence or alteration of eye structures. We also used the *P. tepidariorum*’s autofluorescence to explore the mutant phenotypes and characterize different parts of the eyes of the spider affected after the CRISPR‐KO.^[^ ^31^, ^32^ ^]^

**Figure 2:** CRISPR knock‐out of the eye development gene *sine oculis* (*so*). a) Spider eyes reflect evolutionary adaptations. Spiders like Theriidae and Araneidae rely on silk‐trapping for food, while Saltacidae have large anterior eyes for visual hunting. Comparisons with troglomorphic groups (with total eye reduction), such as *C. isrealensis*, identified *so* as a key gene for eye development.^[^ ^25^, ^26^, ^29^, ^30^ ^]^ Spider eyes are classified as lateral (grey) and anterior (red) based on developmental origin. b) CRISPR knock‐out of *so* in *P. tepidariorum* produced mutations, ranging from major eye loss (*mt*‐1, *mt*‐4) to partial loss (*mt*‐2, *mt*‐3). In *mt*‐1, most eye structures were absent except the lens, while *mt*‐4 showed a complete loss of eye structures. In *mt‐*2, the tapetum and lateral eye structures were missing, though some opsins remained in the anteromedial eyes. Fluorescent microscopy (*) showed that the cuticle remained intact. Notably, the cuticle covering the lens developed normally in all mutants, suggesting that its formation is *so*‐independent. *mt*‐3 showed asymmetry, with one anterior eye lost and the other developed correctly (scale bars: 2 mm). The model in the lower right combines lateral and anterior eye structures to guide understanding of the affected parts.

RETRACTED

It could be confirmed that the CRISPR‐KO impacted the development of all eyes of the respective spider supporting the previously described role of *so* (Figure S1A).^[^ ^25^ ^]^ While most embryos lacked any visual phenotype, some did display irregular eye development not observed in the wild type counterpart. The most conspicuous phenotype was the loss of all the eyes or the anterior‐medial eyes, both of which can clearly be seen using a stereomicroscope (Figure 2b). Strikingly, mutations at the lateral eyes also lacked the tapetum altogether with other structures. The only structure of the eye that was never affected was the lens, suggesting a different developmental origin. To further explore the phenotypic effect, we used the green autofluorescence of *P. tepidariorum* when exposed to blue light to better visualize the gene editing effects (Figure 2b). In some cases, it was noticed that the red‐brown ring preceding the formation of the eyes was either not formed or lost its shape where it should have been developed. This finding supports that the function of the gene *so* is to turn on or off a developmental pathway relevant for the expression of genes involved in eye development of all the spider eyes, including eye patterning genes. Notably, this confirmed that *so* is an important gene for eye development, and affecting its expression would lead from partial to total deformation of all the eyes of the spiders (Figure S1B).^[^ ^25^, ^29^ ^]^

### CRISPR‐KO Genotyping

Electrophoresis (Figure S2) and Sanger sequencing (Figure S3) were used to evaluate the genetic modification efficiency of our approach. The first was used to reveal the size and number of bands, which indicated the quality of the amplifications. The sequences were analyzed using the Synthego‐Inference of CRISPR Edits (ICE) analysis tool,^[^ ^33^ ^]^ which is a bioinformatics software specially designed to identify and characterize DNA Indels, variations at the DNA sequence caused after CRISPR cleavage. The results showed that CRISPR cut near the target gRNA site but generated different Indels. Because spiders were virgins at the time of microinjection and only fertilized post‐microinjection, our results suggest that CRISPR‐induced cleavage occurred at fertilization and early cell cleavages. If there was only one cell or a prolonged syncytial stage, we would have expected a mutation rate of 50% or higher. Instead, we observed mutations with a rate of less than 50% as early cellularization might have occurred, and the CRISPR‐Cas9 ribonucleic complex would have to pass through cell membranes. The mutant samples showed various types of mutations in their DNA sequences, ranging from partial to total cleavage (Figures S4–S7). However, most of the samples showed chimeric mutations, which are typical for CRISPR‐mediated editing. Regarding microinjection efficiency, 90 to 100 nymphs per egg sac were sampled from 59 egg sacs, four of which carried mutant offsprings. Among the sampled offspring, 12 exhibited phenotypic variations, five of which were confirmed by sequencing to carry a mutation induced by CRISPR at the target site (Table S1). Low mutation frequencies per individual are commonly observed in species with high offspring numbers, especially when microinjection is delivered directly to the parent.^[^ ^10^, ^34^, ^35^, ^36^ ^]^ We also observed that only the first egg sacs laid by microinjected spiders contained mutant offspring. Future approaches should account for the ovulation timing to optimize the ribonucleoprotein uptake by the eggs as they are more likely to absorb proteins during this stage.^[^ ^19^ ^]^

RETRACTED

### CRISPR‐Induced Knock‐In (KI)

Having successfully established CRISPR‐Cas9‐based genetic engineering in spiders, we next aimed to functionalize its spider silk and chose one of several major ampullate spidroins (MaSp), namely MaSp2. Orb weaving spiders produce up to seven different types of silk, which differ in their composition and mechanical properties. The most investigated spider silk type is the major ampullate silk, and MaSps represent the main part of major ampullate silk fibers used as a lifeline and as frame‐forming fibers of an orb web.^[^ ^37^, ^38^, ^39^ ^]^ The protein composition of major ampullate silk has been well described, and the two major protein components are MaSp1, a protein with low proline residue content, and MaSp2, a protein with high proline residue content,^[^ ^40^, ^41^ ^]^ which together are held responsible for most of the mechanical traits of the major ampullate silk. The maximum strength of major ampullate silk fibers is up to 1.7 GPa, which is in the range of synthetic high‐tech materials. However, such spider silk fibers have much higher toughness and extensibility than, e.g., Kevlar and carbon fibers based on a combination of high tensile strength and elasticity.^[^ ^42^ ^]^ All MaSps comprise a large central domain of repeated sequence motifs flanked by non‐repetitive (NR) domains, consisting of 100–140 amino acids, which are highly conserved between different spider species and silk types. The flanking NR amino terminal (NTD) and carboxyl terminal domains (CTD) regulate MaSp assembly during storage and along fiber spinning, while the central repetitive sequences are responsible for the mechanical properties of the fibers.^[^ ^37^, ^43^, ^44^, ^45^, ^46^ ^]^

We targeted the linker region connecting the last repetitive motif of the core domain and the CTD of MaSp2 of *P. tepidariorum* for the KI of the monomeric red fluorescent protein (mRFP) because this linker sequence is conserved between spiders but predicted to not participate in the assembly of the protein. The microinjected mRFP sequence, within the pEX‐A258 vector, was designed to be flanked by the linker‐CTD sequence upstream and downstream of the target region of MaSp2. Additionally, it contains the gRNA target regions to be cleaved and linearized when microinjected together with the CRISPR:gRNA solution (mRFPplasmid 100 ng µL^−1^, Cas9: 1 µg µL^−1^, gRNA: 1 µg µL^−1^). Therefore, if inserted successfully at the linker region before the CTD, it was assumed to cause red fluorescence of the major ampullate silk fibers. Indeed, the generated mutant silk revealed red fluorescence (Figure 3a).

**Figure 3:** KI of an mRFP sequence in spider major ampullate silk using CRISPR‐Cas9. a) Comparison of wt and mRFP‐modified major ampullate silk fibers rolled on a capillary glass (scale bars: 550 µm). b) Strong red fluorescence can also be seen in the major ampullate gland (scale bar: 277 µm). c i) The genomic implementation of mRFP into the major ampullate silk was confirmed by amplifying the mRFP DNA sequence extracted from the spider's leg. Only those spiders with red fluorescent silk (scale bar: 138 µm) showed the mRFP sequence‐derived signal in the agarose gel. C ii) Total‐RNA was extracted from the glands, reverse‐transcribed, and subjected to R‐TqPCR and a melting curve analysis showing a peak at 83°C and 87°C based on a small and a large, amplified fragment.

RETRACTED

The respective individuals showing red‐fluorescent silk were anesthetized with CO_2_ to remove a leg for DNA genotyping. The mRFP‐DNA was amplified, and the presence of the amplicon was observed using electrophoresis. The major ampullate silk gland of those spiders with amplified mRFP‐DNA were then dissected, and its RNA amplified (Figure 3b,c, i). The spiders carrying the mutation were then reproduced, and the offspring were further characterized. The screening of the offspring was conducted at early stages because the exoskeleton is not pigmented and is translucent. Some offspring exhibited a red fluorescence within the opisthosoma resembling the shape of a silk gland (Figure S8). Based thereon, we have been able to establish a stable spider line.

Unfortunately, it was not possible to identify the type of gland just by microscopy without dissection. The remaining offspring were allowed to grow to dissect the glands at an adult stage, and it could be confirmed that the red fluorescence was in the major ampullate gland. Total RNA was extracted and analyzed using RT‐qPCR and melting curves (Figure 3c, ii). The results indicated that the mRFP sequence was expressed, and the red fluorescence could be linked to the transcription of the mRFP‐DNA. The cDNA was used for RT‐qPCR, and it was analyzed using Sanger sequencing, confirming the correctness of the mRFP sequence (Figure S9). Examination using a fluorescence microscope located the red fluorescence at the tail of the major ampullate gland (Figure 4). Thus, CRISPR‐Cas9 can be used to KI a desired sequence into that of spider silk proteins, allowing the functionalization of the corresponding silk fibers.

**Figure 4:** mRFP fluorescence within the major ampullate gland. a) Red fluorescence could be detected in the offspring of the KO mutant spiders in the major ampullate gland (scale bar: 277 µm). b) The cartoon recreates the major structures of the major ampullate silk gland: tail, sac, and spinning duct. c) The highest fluorescence intensities could be observed between the tail and the sac (scale bar: 140 µm).

## Conclusion

We have established a protocol for implementing CRISPR‐based KO and KI gene editing in spiders, which differs from protocols used for other organisms. Desired phenotypes could be produced with an efficiency of ∼6%–7% of the egg sacs carrying the respective mutation. The results confirmed that a mutation at the coding sequence of the chosen KO gene *so* impaired eye development of the spider. After successfully establishing the technology in spiders, the insertion of mRFP in their silk was possible when co‐injected with a donor sequence. The ability to employ CRISPR gene engineering in spider silk holds significant promise for research concerning material sciences.^[^ ^8^, ^47^ ^]^ The here used MaSp*2*, one of the main components of the major ampullate silk fiber not known to have a major role during spider development, served as a first model for designing silk fibers with new features that help us to understand their functionalization attaining future applications. However, the CRISPR‐Cas9 technology in spiders also enables evolutionary and developmental studies, particularly understanding early cell developmental stages of cell‐to‐cell communication.^[^ ^22^ ^]^ As an example, CRISPR‐KO experiments can be used to characterize transcription changes after gene KO, helping to understand deep homology and evolution of co‐opted pathways across arthropods.

RETRACTED

## Conflict of Interests

The authors declare no conflict of interest.

## Supporting information



Supporting Information

## Data Availability

The data that support the findings of this study are available from the corresponding author upon reasonable request.
